The article "Harnessing Mucor spp. for Xylanase Production: Statistical Optimization in Submerged Fermentation Using Agro-Industrial Wastes" was published in 2022. Journal: Biomed Res Int.

# Harnessing *Mucor* spp. for Xylanase Production: Statistical Optimization in Submerged Fermentation Using Agro-Industrial Wastes

**DOI:** 10.1155/2022/3816010

**Published:** 2022-04-20

**Authors:** Amal A. Al Mousa, Nageh F. Abo-Dahab, Abdallah M. A. Hassane, Abd El-Rahman F. Gomaa, Jana A. Aljuriss, Noura D. Dahmash

**Affiliations:** ^1^Department of Botany and Microbiology, College of Science, King Saud University, Riyadh, P. BOX 145111, ZIP, 4545, Saudi Arabia; ^2^Botany and Microbiology Department, Faculty of Science, Al-Azhar University, Assiut 71524, Egypt; ^3^King Saud University, Vice Rectorate for Graduate Studies and Scientific Research, Deanship of Scientific Research, Research Assistant Internship Program, Saudi Arabia

## Abstract

Xylan is the primary hemicellulosic polymer found in lignocellulosic agricultural wastes and can be degraded by xylanase. In the current research, *Mucor circinelloides* and *M. hiemalis* were tested for their ability to produce xylanase from tangerine peel by submerged fermentation. Experiments on five variables were designed with Box–Behnken design and response surface methodology. Analysis of variance was exercised, the xylanase output was demonstrated with a mathematical equation as a function of the five factors, and the quixotic states for xylanase biosynthesis was secured. In addition, xylanase was partially purified, characterized, and immobilized on calcium alginate beads. The optimum parameters for xylanase production by *M. circinelloides* and *M. hiemalis* were consisted of incubation temperature (30 and 20°C), pH value (9 and 7) incubation period (9 and 9 days), inoculum size (3 and 3 mL), and substrate concentration (3 and 3 g/100 mL), respectively. *M. circinelloides* and *M. hiemalis* demonstrated the highest xylanase activities after RSM optimization, with 42.23 and 35.88 U/mL, respectively. The influence of single, interchange, and quadratic factors on xylanase output was investigated using nonlinear regression equations with significant *R*^2^ and *p* values. The partial purification of *M. circinelloides* and *M. hiemalis* xylanase yielded 1.69- and 1.97-fold purification, and 30.74 and 31.34% recovery with 292.08 and 240.15 U/mg specific activity, respectively. Partially purified xylanase from *M. circinelloides* and *M. hiemalis* demonstrated the highest activity at neutral pH and 60 and 50°C, respectively. The immobilized *M. circinelloides* and *M. hiemalis* xylanase retained 84.02 and 79.43% activity, respectively. The production of xylanase from *M. circinelloides* and *M. hiemalis* utilizing RSM is deemed profitable for the decomposition of the agro-industrial wastes.

## 1. Introduction

Biotechnological processes on filamentous fungi have enabled the industrial utilization of their ability to produce valuable enzymes due to their ease of propagation and increased production of extracellular enzymes with specific characteristics such as stability over a wide range of pH and temperature [1–3].

The article "Harnessing Mucor spp. for Xylanase Production: Statistical Optimization in Submerged Fermentation Using Agro-Industrial Wastes" was published in 2022. Journal: Biomed Res Int.

The class Zygomycetes, order Mucorales, including the genus *Mucor*, are mainly saprobic fungi that can grow well on various agro-industrial wastes with the potential to produce extracellular hydrolytic enzymes that can be utilized in a variety of industrial applications [4].

The elevated dilation of agricultural junks apostasy has resulted in the cumulation of significant amounts of lignocellulosic wastes across the globe [5]. Lignocellulosic plant biomass mainly comprises hemicellulose, cellulose, and lignin [6]. The most crucial hemicellulosic heteroglycan is xylan, which contains a long chain of *β*-1,4-linked xylopyranose monomers and comprises a significant renovatable biocluster containing up to 20-35% of the dry mass of agricultural residues [5, 7]. Two main xylanolytic enzymes (endo-*β*-1,4-xylanases and exo-*β*-1,4-xylanases) are a candidate to degrade xylan into xylose and xylooligomers [8]. Xylanase is included in various industrial applications like animal food, feed, biobleaching, biofuel, pharmaceutics, textile [9], and juice clarification [10].

The amount of fungal enzyme manufactured is determined by the conditions of the fermentation process and the need to optimize these conditions for low enzyme output cost [11]. The fungal enzyme manufacturing is prevalently implemented by submerged or solid-state fermentation [12]. Submerged fermentation, utilized in 90% enzyme industry, occurs in the presence of water excess, providing a soft handling and best control [13, 14]. Immobilization of enzymes and entrapment of enzymes in polymers such as alginate eliminate the need to isolate the enzyme from the outcome solution, facilitate enzyme recycling, enable repetitive and continuous use, and control enzyme activity [15–18].

This study aimed to evaluate the production of high-value xylanase by *Mucor* spp. using agro-industrial by-products as a cheap substrate in submerged fermentation conditions. The optimization of xylanase production, as well as characterization and immobilization of partially purified xylanase, was investigated.

## 2. Materials and Methods

### 2.1. Tested Fungi

*Mucor circinelloides* AUMC 6696.A (Accession no. MT509983) and *M. hiemalis* AUMC 6031 (Accession no. MT365791) [19] were utilized in the current search for xylanase production. Pure cultures were kept in potato dextrose agar (PDA) tubes and preserved at 4°C for further use.

The article "Harnessing Mucor spp. for Xylanase Production: Statistical Optimization in Submerged Fermentation Using Agro-Industrial Wastes" was published in 2022. Journal: Biomed Res Int.

### 2.2. Enzymes Preliminary Screening

#### 2.2.1. Screening on Agar Plates

Czapekʼs agar medium (g/L: KH2PO_4_, 1; NaNO_3_, 2; MgSO_4_.7H_2_O, 0.5 and CaCl_2_.2H_2_O, 0.5) was supplemented with 10 g/L of xylan powder as a carbon source for xylanase production. The pH was set to 7, and the impregnated plates were preserved at 28 ± 2°C for five days and then screened for enzymes production [20]. After immersing the cultured agar plates in iodine solution for 15 minutes, they were examined for the presence of a clear zone.

#### 2.2.2. Screening by Submerged Fermentation (SmF)

Pomegranate peel, tangerine peel, and wheat straw were desiccated at 65°C for 24 h, then squelched to grist, and used as substrates (10 g/L) in Czapekʼs mineral salts broth. The broth containing flasks was adjusted to pH 7 and autoclave sterilized. The strains' spore suspensions (10^7^ spores/mL) were utilized to inoculate 250-mL flasks holding 100 mL submerged broth. The impregnated flasks were preserved at 28 ± 2°C for seven days on both shaking and static conditions. Subsequently, broth media were centrifuged, and supernatants were maintained for further enzymatic analysis.

#### 2.2.3. Quantitative Screening of Xylanase

Xylanase efficiency was measured according to Miller [21]. In addition, 0.5 mL enzyme supernatant was added to 0.5 mL xylan (1% w/v) in acetate buffer, and the mixture was incubated at 50°C for 30 min. Afterward, the interaction was intercepted by appending 1 mL of 3,5-dinitrosalicylic acid reagent and incubated at 100°C for 10 min. After cold dishing, the absorbance was measured at 570 nm using a spectrophotometer (Jenway 7315, UK). The amount of reducing sugars was determined using xylose as a standard for plotting the calibration curve. All the tests were carried out three times, and the outputs were expressed as an average value. A unit of the enzyme was acquainted as the quantity of the enzyme per one mL required to release one *μ*mol of reducing sugar from a substrate per 60 seconds under the optimum trial conditions [22].

### 2.3. Optimization of Enzymatic Productivity under Submerged Fermentation (SmF)

Response surface methodology (RSM) tactic using Box–Behnken design (BBD) was exercised to determine the optimum factors for boosted xylanase production, including A, temperature; B, pH; C, incubation period; D, inoculum size; and E, substrate concentration (Table 1). Forty-six experiments with the central points were employed to satisfy the polynomial pattern established on a Box–Behnken design (BBD, 5 variables) attained by Minitab 19® software (Version19.1.1.0. LLC). At three-level and five factors, experimental BBD was examined, and the number of the tests (*N*) was determined corresponding to the subsidiary equation:

(1) $$\begin{array}{c} N=2k*\left(k-1\right)+C0 \end{array}$$

where *k* is the digit of factors and *C*0 is the digit of central points equal to 6.

The article "Harnessing Mucor spp. for Xylanase Production: Statistical Optimization in Submerged Fermentation Using Agro-Industrial Wastes" was published in 2022. Journal: Biomed Res Int.

The impact of variables on the simulation (*Y*) was evaluated by utilizing a second-order polynomial equation to determine the quixotic states of the xylanase biosynthesis.

(2) $$\begin{array}{c} Y=\beta_{0}+\beta_{1}A+\beta_{2}B+\beta_{3}C+\beta_{4}D+\beta_{5}E+\beta_{11}A^{2}+\beta_{22}B^{2}+\beta_{33}C^{2}+\beta_{44}D^{2}+\beta_{55}E^{2}+\beta_{12}AB+\beta_{13}AC+\beta_{14}AD+\beta_{15}AE+\beta_{23}BC+\beta_{24}BD+\beta_{25}BE+\beta_{34}CD+\beta_{35}CE+\beta_{45}DE \end{array}$$

where *Y* (response variable); *β*_0_ (intercept); *β*_1_, *β*_2_, *β*_3_, *β*_4_, and *β*_5_ (linear coefficients); *β*_11_, *β*_22_, *β*_33_, *β*_44_, and *β*_55_ (square coefficients); *β*_12_, *β*_13_, *β*_14_, *β*_15_, *β*_23_, *β*_24_, *β*_25_, *β*_34_, *β*_35_, and *β*_45_ (interaction coefficients); and *A*, *B*, *C*, *D*, *E*, *A*^2^, *B*^2^, *C*^2^, *D*^2^, *E*^2^, AB, AC, AD, AE, BC, BD, BE, CD, CE, and DE (levels of independent variables). The corresponding coefficients of variables, interaction variables, and contour graphs were obtained by Minitab 19® software. By analyzing the regression equation and constructing the response plots, the ideal values of the tested variables were secured. The coefficient of limitation *R*^2^ was used to express the fineness of profit of the polynomial equation, and the (*F*) test was used to determine its statistical significance level.

### 2.4. Partial Purification of Xylanase from *Mucor* Strains

After the incubation period under optimum conditions, the contents of the broth culture were centrifuged, and the supernatant was utilized for enzyme assay. Xylanase activity and protein concentration were measured in the supernatant according to Miller [21] and Lowry et al. [23], respectively, utilizing the standard of bovine serum albumin to generate the calibration curve spectrophotometrically at 750 nm.

Crude enzyme solution was partially purified by precipitation using cold acetone. Precooled acetone (-20°C) was subjoined to the enzyme solution until the volume ratio between enzyme solution and acetone reached 1 : 1; 1 : 2; 1 : 3; 1 : 4, and 1 : 5 (v/v). The solution was left at -20°C overnight to allow protein precipitation. The precipitates were gathered by centrifugation at 10000 rpm for 15 min and resuspended in a small volume of (sodium citrate buffer, pH 4.8, 0.05 M). These samples were used for determining the activity of xylanase, purification factor, and enzyme recovery yield [24]. Protein was estimated, and suitable precipitants for characterization were selected. The following equations were used to calculate the partially purified xylanase's specific activity, yield, and purification fold.

(3) $$\begin{array}{c} \text{Specific activity}\left(\text{U}/\text{mg}\right)=\frac{\text{Total activity}}{\text{Total protein}},\\ \text{Yield}\left(\%\right)=\frac{\text{Total units in partially purified enzyme}\times 100\%}{\text{Total units in crude enzyme}},\\ \text{Purification fold}=\frac{\text{Specific activity of partially purified enzyme }}{\text{Specific activity of crude enzyme}}. \end{array}$$

The article "Harnessing Mucor spp. for Xylanase Production: Statistical Optimization in Submerged Fermentation Using Agro-Industrial Wastes" was published in 2022. Journal: Biomed Res Int.

### 2.5. Characterization of Partially Purified Xylanase

The optimum temperature for partially purified xylanase activity was determined to be in the range of (30-90°C), and the thermal stability was determined after premaintaining the enzyme at each temperature degree for one hour before screening. Ideal pH estimation was carried out at optimum temperature utilizing various buffers with values (3-11), and the pH stability was assessed after preserving these pH values for 1 h before the screening. In addition, xylanase activity was estimated after maintaining the enzyme with different metal ions (10 mM of K^+^, Mg^2+^, Ba^2+^, and Ni^2+^) for 1 h at optimum temperature and pH. Xylanase activity was assessed after processing with diverse detergents comprising tween 80 and 20 at concentrations of 1 and 5% v/v, urea (1 and 5% w/v), and Na_2_CO_3_ (50 and 75 mM) compared to control (100% activity) [25, 26].

### 2.6. Immobilization of Xylanase

The immobilization of partially purified xylanase was performed by combining enzyme solution with an equal volume of 3.0% sodium alginate solution. Calcium alginate beads were formalized by adding the mixture drop-wise in 0.2 M CaCl_2_ at 4°C. Calcium alginate beads were rinsed by double-distilled H_2_O to remove unstriated enzyme units. Then, the beads were desiccated and stored in phosphate buffer. The entrapped beads were activated using glutaraldehyde for covalent binding of xylanase onto the beads [27], and the assay of free and immobilized xylanase was performed. The immobilization yield was assayed according to the equation [28].

(4) $$\begin{array}{c} \text{Immobilization yield}\left(\%\right)=\frac{Ai-\text{Af}}{A\text{f}}\times 100, \end{array}$$

where *Ai* is the immobilized enzyme activity and *Af* is the free enzyme activity.

#### 2.6.1. Scanning Electron Microscopy

A scanning electron microscope (JEOL JSM 5400, Japan) was utilized to examine the outer surface forms of calcium alginate beads before and after xylanase immobilization.

### 2.7. Data Analysis

All tests and measurements were repeated three times. Using the SPSS, software program (version No. 16), and one-way ANOVA, the values were expressed as the mean ± SD at the 0.05 significance level.

The article "Harnessing Mucor spp. for Xylanase Production: Statistical Optimization in Submerged Fermentation Using Agro-Industrial Wastes" was published in 2022. Journal: Biomed Res Int.

## 3. Results

### 3.1. Preliminary Screening of Xylanase Production

The preliminary screening for extracellular fungal xylanase revealed that both *M. circinelloides* and *M. hiemalis* had a high potential to produce xylanase qualitatively on a solid assay medium. They were then quantitatively assayed under SmF and produced 21.77 and 15.28 U/mL, respectively, on the tangerine peel as a substrate under static condition (Table 2).

### 3.2. Response Surface Methodology for Optimization of Xylanase Production

Table 1 shows the independent factors with their competent levels employed in optimization of xylanase output, while BBD of the independent factors along with predicted as well as experimental values are depicted in Table 3. The production of xylanase by *M. circinelloides* was predicted using the following equation:

(5) $$\begin{array}{c} Y\left(U/mL\right)=16.6+4.495A-15.60B-0.51C-1.73D+2.01E-0.01559A^{2}+0.5968B^{2}-0.0546C^{2}-0.7799D^{2}+0.3562E^{2}-0.1042AB-0.3331AC+0.0052AD-0.3537AE+1.397BC+0.010BD+0.443BE+0.820CD+0.330CE+0.150DE \end{array}$$

While the production of xylanase by *M. hiemalis* was predicted by the following equation:

(6) $$\begin{array}{c} Y\left(U/mL\right)=51.0+0.236A-7.99B+4.59C-8.71D+2.81E+0.03131A^{2}+0.828B^{2}+0.020C^{2}+0.066D^{2}-0.164E^{2}+0.0196AB-0.2217AC-0.1815AD-0.1753AE-0.412BC-0.031BD-0.727BE+1.284CD+0.505CE+1.268DE \end{array}$$

The highest xylanase activity of both *M. circinelloides* (42.23 U/mL) and *M. hiemalis* (35.88 U/mL) was obtained from runs No. 27 to 46, respectively. The run No. 27 for *M. circinelloides* consisted of incubation temperature (30°C), pH value (9), the incubation period (9 days), inoculum size (3 mL), and substrate concentration (3 g/100 mL). In comparison, the run No. 46 for *M. hiemalis* consisted of incubation temperature (20°C), pH value (7), the incubation period (9 days), inoculum size (3 mL), and substrate concentration (3 g/100 mL).

Analysis of variance (ANOVA) for the xylanase quadric model of *M. circinelloides* and *M. hiemalis* is shown in Tables 4 and 5. Model terms with a *p* value <0.05 were deemed significant. The model *F* value of 58.10 and 17.59 for *M. circinelloides* and *M. hiemalis*, respectively, indicated that the model is significant. Values of “Prob > *F*” <0.05 pointed model terms are significant. In this case, *A*, *B*, *C*, *E*, *A*^2^, *B*^2^, *D*^2^, *E*^2^, AB, AC, AE, BC, BE, CD, and CE are significant model terms for *M. circinelloides*, while for *M. hiemalis*, *A*, *B*, *C*, *D*, *E*, *A*^2^, *B*^2^, AC, AD, AE, BE, CD, CE, and DE are significant model terms. The “Lack of Fit *F*-value” of 0.83and 0.58for *M. circinelloides* and *M. hiemalis*, respectively, indicated that the lack of fit is insignificant concerning the pure error. Nonsignificant lack of fit is proper for the model to be convenient. The resulted multiple correlation coefficient (*R*^2^ = 0.9789 for *M. circinelloides* and *R*^2^ = 0.9336 for *M. hiemalis*) that nigh to 1 betokened preferable interconnection between experimental and predicted values and elucidated the model accuracy with upgrade response.

The article "Harnessing Mucor spp. for Xylanase Production: Statistical Optimization in Submerged Fermentation Using Agro-Industrial Wastes" was published in 2022. Journal: Biomed Res Int.

Contour plots explained the relationship between parameters and defined each factor's optimum scale for xylanase efficiency by *M. circinelloides* (Figures 1(a)–1(j)) and *M. hiemalis* (Figures 2(a)–2(j)). The response surface plot constructed any two variables, while other variables were maintained at their optimal level. Contour plots of xylanase activity by *M. circinelloides* revealed significant interactions between incubation temperature with pH, incubation period, and substrate concentration; pH with incubation period and substrate concentration; and incubation period with inoculum size and substrate concentration. In contrast, contour plots of the interactions between incubation temperature with incubation period, inoculum size, and substrate concentration; pH with substrate concentration; incubation period with inoculum size and substrate concentration; and inoculum size with substrate concentration significantly influenced xylanase production by *M. hiemalis*. The remaining interactions insignificantly influenced xylanase production.

### 3.3. Partial Purification of Xylanase

Extracellular xylanase from *M. circinelloides* and *M. hiemalis* was partially purified from broth cultures by using different acetone concentrations. The highest xylanase activity (11.89 and 10.73 U/mL from *M. circinelloides* and *M. hiemalis*, respectively) was obtained via crude filtrate precipitation with acetone at ratio 1 : 4 (Table 6). Xylanase purification resulted in 1.69-fold purification and 30.74% xylanase recovery with a specific activity of 292.08 U/mg from *M. circinelloides*, while in 1.97-fold purification, 31.34% recovery with a specific activity of 240.15 U/mg was obtained from *M. hiemalis* xylanase (Table 7).

### 3.4. Characterization of Partially Purified Xylanase

*M. circinelloides* partially purified xylanase was highly active at 60°C (total activity 100%) and decreased gradually at 50-30°C and 70-90°C, while xylanase activity of *M. hiemalis* was highly active at 50°C (total activity 100%) and decreased gradually at 40-30°C and 60-90°C. The relative xylanase stability from both *M. circinelloides* and *M. hiemalis* was high at 30°C and decreased in the range of 40-90°C (Figures 3(a) and 3(b)). Furthermore, partially purified xylanase from both strains had the highest activity and stability (100%) at pH 7.0, and then, at higher or lower pH values, activity and stability of xylanase were reduced (Figures 3(c) and 3(d)).

The article "Harnessing Mucor spp. for Xylanase Production: Statistical Optimization in Submerged Fermentation Using Agro-Industrial Wastes" was published in 2022. Journal: Biomed Res Int.

After incubation with 10 mM K^+^, Mg^2+^, Ba^2+^, and Ni^2+^, xylanase activity of both strains decreased with the exception of K^+^, which increased *M. hiemalis* xylanase activity by 40.34% compared to the control, while stability increased except for Ba^2+^ with *M. circinelloides* enzyme and K^+^ and Mg^2+^ with *M. hiemalis* enzyme. Detergents including Tween 80, Tween 20, urea, and Na_2_CO_3_ at low concentrations of 1%, 1%, 1%, and 50 mM, respectively, reduced *M. circinelloides* and *M. hiemalis* partially purified xylanase activity. In contrast, there was a significant increase in activity and decreased stability at high concentrations of the tested detergents, except urea, which decreased *M. hiemalis* partially purified xylanase activity at its applied high concentration (5%) (Table 8).

### 3.5. Xylanase Immobilization and Scanning Electron Microscopy

*M. circinelloides* enzyme had an immobilization yield of 84.02%, while *M. hiemalis* enzyme had a yield of 79.43% (Table 9). A scanning electron microscope was utilized to investigate the surface superficial of calcium alginate beads together and without entrapped xylanase (Figure 4). The vents of calcium alginate beads were examined in the micrographs of calcium alginate beads without entrapped xylanase, whereas together with xylanase, the vents were coated with intense molecule xylanase.

## 4. Discussion

Fungi play an excellent source for the production of various beneficial enzymes. Xylan represents the principal hemicellulosic xylopolymer found in plant cell walls. The biodegradation of xylan functions as an essential role of plant materials natural [29]. In this research, *M. circinelloides* and *M. hiemalis* were investigated as potential sources for producing xylanase.

Many fungi were proven to have multiple xylanase forms and can efficiently breakdown xylan. In addition, the substrate type influenced the concentration and number of various expressed forms of xylanase [30, 31]. On the contrary, the substrate installation and growth factors affect the fungal growth and the biosynthesis of enzymes. Therefore, there is an urgent need to modify the biosynthesis of the enzymes by optimizing fungal production.

In the current research, the low *p* values, which are attained by the *F* test, and high *R*^2^ values indicated that the employed model attained a high significance, and its sufficiency was confirmed [32]. For xylanase production on wheat bran by solid-state fermentation by *M. indicus* and *M. hiemalis* using RSM, the optimum temperatures were 40.0 and 43.4 °C, respectively, and 51.3 and 53.2 h for incubation time, respectively, while the highest xylanase activities were 43.1 and 43.8 U/g for *M. indicus* and *M. hiemalis*, respectively [33]. Atalla et al. [34] reported a maximum xylanase activity from *A. oryzae* (0.37 U/mL) by utilizing rice straw waste, while orange peel exhibited low xylanase production (0.17 U/mL). Cui and Zhao [35] highlighted the magnitude of the substrate concentration for xylanase biosynthesis, where the enzyme activity by *Penicillium* sp. WX-Z1 demonstrated a gradual rise in wheat bran concentration. Statistical analysis of xylanase production from *Penicilliumoxalicum* ZH-30 by RSM showed that the linear, quadric terms and initial pH and temperature interaction significantly impacted the optimal conditions for raised xylanase biosynthesis at pH 7.38 and temperature 31.1°C. Under optimal conditions, the portended and experimented xylanase activities were 14.33 and 14.50 U/mL, respectively [36].

The article "Harnessing Mucor spp. for Xylanase Production: Statistical Optimization in Submerged Fermentation Using Agro-Industrial Wastes" was published in 2022. Journal: Biomed Res Int.

Box–Behnken design statistical analysis by Cao et al. [37] demonstrated that the linear and quadric terms of cultivation time, pH, and substrate concentration variables significantly affected xylanase production by *Aspergillus niger*AN-13 using wheat bran under submerged fermentation. In submerged fermentation with corncob, *Aspergillus niger* KIBGE-IB36 was found to be a high producer of xylanase [38] and different spectra of xylanase synthesis using wheat bran, rice husk, orange peel, and pomegranate peel [5]. RSM method by Azzouz et al. [39] reported a 65.01% increase in xylanase output by *Aspergillus niger* strain BG on 84% humidified wheat bran with a pH of 2.5 at 37°C and incubation for 66 h. Statistical analysis of xylanase output by *Aspergillus foetidus* in submerged fermentation with soybean scraps revealed that variables pH and the interaction of pH and temperature influenced xylanase biosynthesis, with good xylanase activity (13.98 U/mL) at pH 7.0, 28 °C, and 120 rpm for 168 hours [40]. Response surface methodology by Ramanjaneyulu and Rajasekhar [41] for maximal production of xylanase (4560 U/mL) by *Fusarium* sp. BVKT R2 demonstrated that the optimal conditions were sorbitol 1.5%, yeast extract 1.5%, pH of 5.0, temperature of 32.5 °C, and shaking of 175 rpm.

High temperature increases the solubility of reactants and products by decreasing viscosities, resulting in faster hydrolysis [42], and prolonged energetic existence would fabricate enzymes convenient for promoted and active biomass diversion. Therefore, thermostability is the most substantial property for the enzyme used under extreme bioprocessing conditions to be efficient [8]. RSM optimization of xylanase yield by *Aspergillus niger* 3-fold and 1.41-fold purification was attained with about 6.2% yield, and the highest activity of the purified xylanase was observed at pH 6 and 50°C. The produced xylanase exhibited high thermal and pH stability, with more than 90% residual activity between 30 and 40°C and pH 3-9 after incubation of 24 h, with half-lives of 30 min at 50 and 60°C [43]. Liet al. [36] reported a temperature range of 50-60°C suitable for the industrial application of xylanase from *P. oxalicum* ZH-30. Supplementation of Tween 80 as additional surfactant improved (72.4 ± 1.42 U/g) the titer of xylanase on sugarcane bagasse by *T. viride*-IR05 [44]. Regarding xylanase immobilization, the formation of an ionic bond of Ca^2+^ with carboxylate groups of sodium alginate helm to formulate mechanically firm grids of alginate gel that fulfill the demands for efficient hydrogel systems acting as carriers of bioactive molecules in several industrial applications [45]. Immobilized *Talaromyces thermophilus* xylanase covalently bound by glutaraldehyde to chitosan, chitin, amberlite, duolite, florisil, and gelatin gave immobilization yield of 89.0, 87.8, 89.3, 81.1, 96.2, and 98.8%, respectively [28].

The article "Harnessing Mucor spp. for Xylanase Production: Statistical Optimization in Submerged Fermentation Using Agro-Industrial Wastes" was published in 2022. Journal: Biomed Res Int.

## 5. Conclusion

The present study utilized the response surface methodology via the Box–Behnken design to improve xylanase production by *M. circinelloides* and *M. hiemalis*. The experimental results are consistent with predicted responses. The produced enzyme was partially purified, characterized, and immobilized. The optimum parameters for xylanase production by *M. circinelloides* and *M. hiemalis* consisted of incubation temperature (30 and 20 °C), pH value (9 and 7) incubation period (9 and 9 days), inoculum size (3 and 3 mL), and substrate concentration (3 and 3 g/100 mL), respectively. The partial purification of *M. circinelloides* and *M. hiemalis* xylanase yielded 1.69- and 1.97-fold purification, and the immobilized xylanase retained 84.02 and 79.43% activity, respectively. Response surface methodology was effective and satisfactory and investigated many factors simultaneously. More research is needed to scale up enzyme production for a wide range of applications.

## Figures and Tables

**Figure 1:** Contour plot showing interactions between independent variables (a)–(j) for xylanase activity produced by *M. circinelloides*.

**Figure 2:** Contour plot showing interactions between independent variables (a)–(j) for xylanase activity produced by M*. hiemalis*.

The article "Harnessing Mucor spp. for Xylanase Production: Statistical Optimization in Submerged Fermentation Using Agro-Industrial Wastes" was published in 2022. Journal: Biomed Res Int.

**Figure 3:** Effects of temperature and pH on activity and stability of partially purified xylanase (a) and (c) *M. circinelloides* and (b) and (d) *M. hiemalis*.

**Figure 4:** Scanning electron micrographs (SEM) of calcium alginate beads with and without entrapped xylanase. (a)–(b) Micrographs of calcium alginate beads without enzyme, (c)–(e) micrographs of calcium alginate beads with immobilized xylanase from *M. circinelloides*, and (f)–(h) immobilized xylanase from *M. hiemalis* at magnification scales of 5000× and 10,000×, respectively.

**Table 1:** Box–Behnken design levels of independent factors.

No.	Factor	Variables	Units	Range		
				Minimum	Maximum	Mean
1	A	Temperature	°C	20	40	30
2	B	pH	—	5	9	7
3	C	Incubation period	Day	5	9	7
4	D	Inoculum size	mL	1	5	3
5	E	Substrate concentration	g	1	5	3

**Table 2:** Xylanase production on different substrates under shaking and static conditions.

Substrate	Xylanase activity (U/mL)			
	*M. circinelloides*		*M. hiemalis*	
	Shaking	Static	Shaking	Static
Pomegranate peel	3.26 ± 0.41^b^	2.11 ± 0.31^b^	2.91 ± 0.28^b^	3.73 ± 0.29^b^
Tangerine peel	17.90 ± 0.68^a^	21.77 ± 0.96^a^	13.96 ± 0.13^a^	15.28 ± 0.29^a^
Wheat straw	0.69 ± 0.06^c^	1.32 ± 0.23^b^	2.84 ± 0.52^b^	0.86 ± 0.07^c^

The data were given as averages of three replicates (mean ± SD). Values followed by the different letters are significantly different at *p* < 0.05.

**Table 3:** Box–Behnken design of optimization variables with experimental and predicted xylanase activity of both *M. circinelloides* and *M. hiemalis*.

Run order	Variables					Xylanase activity (U/mL)			
						*M. circinelloides*		*M. hiemalis*	
	A	B	C	D	E	Experimental response	Predicted response	Experimental response	Predicted response
1	40	7	7	5	3	17.73	18.54	17.32	17.49
2	30	7	7	5	1	27.63	27.49	17.23	18.32
3	40	7	7	3	1	31.92	31.24	28.70	28.42
4	20	7	7	3	1	28.62	28.03	30.02	28.82
5	20	9	7	3	3	38.52	38.49	29.69	31.58
6	40	9	7	3	3	23.42	23.39	24.00	24.96
7	30	9	7	3	1	31.67	33.36	28.45	29.76
8	30	9	5	3	3	23.26	22.76	25.07	25.48
9	30	7	7	3	3	27.38	28.56	19.79	23.78
10	30	5	9	3	3	28.45	27.53	32.91	32.16
11	30	5	7	5	3	27.22	26.26	28.12	27.07
12	30	5	7	3	1	32.58	33.81	26.89	27.84
13	30	7	5	3	1	28.37	28.36	27.79	26.20
14	30	9	7	3	5	34.72	34.49	19.54	19.21
15	40	7	7	3	5	15.50	14.68	16.90	16.68
16	30	7	7	3	3	29.28	28.56	23.50	23.78
17	30	5	5	3	3	31.84	30.84	25.32	26.07
18	40	7	5	3	3	25.24	24.05	26.72	26.33
19	20	5	7	3	3	30.02	31.23	34.89	36.26
20	20	7	7	1	3	30.27	29.44	30.93	29.60
21	30	7	9	3	5	33.40	33.82	24.08	24.25
22	30	7	9	3	1	34.81	33.59	26.80	24.94
23	30	7	9	1	3	25.81	25.87	21.11	22.74
24	30	5	7	3	5	28.54	27.85	29.61	28.92
25	30	7	5	3	5	21.69	23.31	16.99	17.42
26	30	9	7	5	3	30.10	29.43	24.49	22.92
27	30	9	9	3	3	42.23	41.80	26.06	24.96
28	30	7	7	3	3	26.89	28.56	23.17	23.78
29	30	7	9	5	3	32.83	32.45	28.78	28.29
30	30	5	7	1	3	26.39	26.31	32.58	31.54
31	30	7	7	1	5	24.91	25.05	17.15	18.30
32	40	5	7	3	3	23.26	24.46	27.63	28.08
33	30	9	7	1	3	29.11	29.32	29.44	27.88
34	20	7	7	5	3	28.95	29.26	30.85	32.15
35	30	7	7	3	3	28.21	28.56	25.40	23.78
36	30	7	7	1	1	28.95	28.66	31.59	33.18
37	40	7	7	1	3	18.64	18.30	31.92	29.46
38	30	7	7	5	5	25.98	26.28	23.09	23.74
39	30	7	5	1	3	23.42	24.56	28.21	30.22
40	30	7	7	3	3	29.86	28.56	25.48	23.78
41	20	7	7	3	5	40.50	39.76	32.25	31.10
42	20	7	5	3	3	22.43	21.66	26.39	24.86
43	40	7	9	3	3	17.56	18.59	18.47	20.24
44	30	7	7	3	3	29.77	28.56	25.32	23.78
45	30	7	5	5	3	17.32	18.03	15.34	15.24
46	20	7	9	3	3	41.41	42.85	35.88	36.52

The article "Harnessing Mucor spp. for Xylanase Production: Statistical Optimization in Submerged Fermentation Using Agro-Industrial Wastes" was published in 2022. Journal: Biomed Res Int.

**Table 4:** ANOVA for the experimental results of xylanase biosynthesis by *M. circinelloides*.

Source	Sum of squares	Degree of freedom	Mean of squares	*F* value	*p* value	Prob > *F*
Model	1608.62	20	80.431	58.10	0.000	Significant
Linear	787.16	5	157.431	113.73	0.000	
A	477.94	1	477.943	345.27	0.000	
B	38.28	1	38.283	27.66	0.000	
C	247.63	1	247.635	178.90	0.000	
D	0.00	1	0.004	0.00	0.958	
E	23.29	1	23.291	16.83	0.000	
Square	237.41	5	47.483	34.30	0.000	
A^2^	21.21	1	21.208	15.32	0.001	
B^2^	49.74	1	49.738	35.93	0.000	
C^2^	0.42	1	0.416	0.30	0.589	
D^2^	84.92	1	84.925	61.35	0.000	
E^2^	17.72	1	17.717	12.80	0.001	
2-way interaction	584.05	10	58.405	42.19	0.000	
AB	17.36	1	17.357	12.54	0.002	
AC	177.51	1	177.513	128.24	0.000	
AD	0.04	1	0.043	0.03	0.862	
AE	200.18	1	200.176	144.61	0.000	
BC	124.96	1	124.958	90.27	0.000	
BD	0.01	1	0.007	0.00	0.945	
BE	12.58	1	12.584	9.09	0.006	
CD	43.01	1	43.015	31.07	0.000	
CE	6.97	1	6.969	5.03	0.034	
DE	1.43	1	1.431	1.03	0.319	
Residual	34.61	25	1.384			
Lack-of-fit	26.62	20	1.331	0.83	0.655	Not significant
Pure error	7.99	5	1.597			
Total	1643.23	45				

*R* ^2^: 0.9789; adjusted *R*^2^: 0.9621; predicted *R*^2^: 0.9282.

**Table 5:** ANOVA for the experimental results of xylanase biosynthesis by *M. hiemalis*.

Source	Sum of squares	Degree of freedom	Mean of squares	*F* value	*p* value	Prob > *F*
Model	1136.70	20	56.835	17.59	0.000	Significant
Linear	489.53	5	97.906	30.30	0.000	
A	219.29	1	219.287	67.86	0.000	
B	60.78	1	60.778	18.81	0.000	
C	31.01	1	31.009	9.60	0.005	
D	88.84	1	88.837	27.49	0.000	
E	89.62	1	89.617	27.73	0.000	
Square	196.46	5	39.292	12.16	0.000	
A^2^	85.58	1	85.581	26.48	0.000	
B^2^	95.63	1	95.630	29.59	0.000	
C^2^	0.05	1	0.055	0.02	0.898	
D^2^	0.61	1	0.611	0.19	0.667	
E^2^	3.76	1	3.762	1.16	0.291	
2-way interaction	450.72	10	45.072	13.95	0.000	
AB	0.61	1	0.614	0.19	0.667	
AC	78.65	1	78.650	24.34	0.000	
AD	52.70	1	52.705	16.31	0.000	
AE	49.17	1	49.172	15.22	0.001	
BC	10.89	1	10.889	3.37	0.078	
BD	0.06	1	0.061	0.02	0.892	
BE	33.83	1	33.827	10.47	0.003	
CD	105.49	1	105.493	32.65	0.000	
CE	16.34	1	16.341	5.06	0.034	
DE	102.97	1	102.966	31.86	0.000	
Residual	80.79	25	3.232			
Lack-of-fit	56.54	20	2.827	0.58	0.823	Not significant
Pure error	24.25	5	4.850			
Total	1217.49	45				

*R* ^2^: 0.9336; adjusted *R*^2^: 0.8806; predicted *R*^2^: 0.7856.

The article "Harnessing Mucor spp. for Xylanase Production: Statistical Optimization in Submerged Fermentation Using Agro-Industrial Wastes" was published in 2022. Journal: Biomed Res Int.

**Table 6:** Precipitation of xylanase produced by *M. circinelloides* and *M. hiemalis* using different acetone concentrations.

Ratio (crude : acetone)	Xylanase activity (U/mL)	
	*M. circinelloides*	*M. hiemalis*
1 : 1	6.92 ± 0.22^c^	5.19 ± 022^c^
1 : 2	5.41 ± 0.27^d^	3.68 ± 0.27^d^
1 : 3	7.25 ± 0.07^c^	5.52 ± 0.07^c^
1 : 4	11.89 ± 0.23^a^	10.73 ± 0.77^a^
1 : 5	9.59 ± 0.34^b^	8.38 ± 0.87^b^

The data were given as averages of three replicates (mean ± SD). Values followed by the different letters are significantly different at *p* < 0.05.

**Table 7:** Summary of specific activity, yield, and purification fold of xylanase produced by *M. circinelloides* and *M. hiemalis*.

Fungal strain	Purification steps	Total activity (U/mL)	Total protein (mg/mL)	Specific activity (U/mg)	Yield (%)	Purification fold
*M. circinelloides*	Culture supernatant	14519.60	86.05	169.09	100	1
*M. hiemalis*		12458.07	102.39	121.74	100	1
*M. circinelloides*	Acetone	4522.52	15.48	292.08	30.74	1.69
*M. hiemalis*	Acetone	3904.07	16.19	240.15	31.34	1.97

**Table 8:** Effects of metal ions and detergents on activity and stability of partially purified xylanase from *M. circinelloides* and *M. hiemalis*.

Metal ions and detergents	Conc.	*M. circinelloides*		*M. hiemalis*	
		Relative activity (%)	Relative stability (%)	Relative activity (%)	Relative stability (%)
Control	0	100.00 ± 0.00	—	100.00 ± 0.00	—
K^+^	10 mM	48.52 ± 0.75	50.55 ± 0.47	140.34 ± 0.34	109.01 ± 1.03
Mg^2+^	10 mM	42.99 ± 0.47	82.08 ± 0.21	96.30 ± 0.44	90.70 ± 2.35
Ba^2+^	10 mM	28.37 ± 0.55	10.10 ± 0.12	77.90 ± 0.69	84.75 ± 1.11
Ni^2+^	10 mM	16.68 ± 0.42	35.12 ± 0.25	38.29 ± 0.96	93.44 ± 1.04
Tween 80	1% (v/v)	53.06 ± 0.83	40.94 ± 0.18	61.76 ± 0.13	35.20 ± 0.49
	5% (v/v)	55.09 ± 0.94	27.99 ± 0.54	72.15 ± 0.11	29.93 ± 0.70
Tween 20	1% (v/v)	61.90 ± 0.28	44.74 ± 0.42	62.33 ± 0.61	47.10 ± 0.68
	5% (v/v)	64.27 ± 0.40	44.57 ± 0.20	65.15 ± 1.05	40.10 ± 1.17
Urea	1% (w/v)	46.58 ± 0.38	37.74 ± 0.59	61.04 ± 0.58	42.13 ± 0.66
	5% (w/v)	59.43 ± 0.80	20.73 ± 0.09	49.89 ± 0.35	27.20 ± 0.67
Na_2_CO_3_	50 mM	30.30 ± 0.89	9.63 ± 0.02	29.37 ± 0.36	22.62 ± 0.22
	75 mM	30.49 ± 0.58	4.44 ± 0.04	40.08 ± 0.82	7.81 ± 0.51

The data were given as averages of three replicates (mean ± SD).

The article "Harnessing Mucor spp. for Xylanase Production: Statistical Optimization in Submerged Fermentation Using Agro-Industrial Wastes" was published in 2022. Journal: Biomed Res Int.

**Table 9:** The immobilization yield (%) of xylanase entrapped in calcium alginate beads.

Fungal strain	*M. circinelloides*	*M. hiemalis*
Yield (%)	84.02 ± 0.63	79.43 ± 0.47

The data were given as averages of three replicates (mean ± SD).

## Data Availability

No data were used to support this study.

## Abbreviations

RSM: Response surface methodology
BBD: Box–Behnken design
ANOVA: Analysis of variance
SmF: Submerged fermentation.
